# Cataract Disease Detection by Using Transfer Learning-Based Intelligent Methods

**DOI:** 10.1155/2021/7666365

**Published:** 2021-12-08

**Authors:** Md Kamrul Hasan, Tanjum Tanha, Md Ruhul Amin, Omar Faruk, Mohammad Monirujjaman Khan, Sultan Aljahdali, Mehedi Masud

**Affiliations:** ^1^Department of Electrical and Computer Engineering, North South University, Bashundhara, Dhaka 1229, Bangladesh; ^2^Department of Computer Science, College of Computers and Information Technology, Taif University, P.O. Box 11099, Taif 21944, Saudi Arabia

## Abstract

One of the most common visual disorders is cataracts, which people suffer from as they get older. The creation of a cloud on the lens of our eyes is known as a cataract. Blurred vision, faded colors, and difficulty seeing in strong light are the main symptoms of this condition. These symptoms frequently result in difficulty doing a variety of tasks. As a result, preliminary cataract detection and prevention may help to minimize the rate of blindness. This paper is aimed at classifying cataract disease using convolutional neural networks based on a publicly available image dataset. In this observation, four different convolutional neural network (CNN) meta-architectures, including InceptionV3, InceptionResnetV2, Xception, and DenseNet121, were applied by using the TensorFlow object detection framework. By using InceptionResnetV2, we were able to attain the avant-garde in cataract disease detection. This model predicted cataract disease with a training loss of 1.09%, a training accuracy of 99.54%, a validation loss of 6.22%, and a validation accuracy of 98.17% on the dataset. This model also has a sensitivity of 96.55% and a specificity of 100%. In addition, the model greatly minimizes training loss while boosting accuracy.

## 1. Introduction

A cataract is a type of eye disease where the eyes look cloudy. A person with cataracts will have frosty or fogged-up vision. A person with cataract eyes faces difficulties reading, driving, and even recognizing another person's face [1]. According to the World Health Organization (WHO), there are approximately 285 million visually impaired individuals worldwide, with 39 million blind people and 246 million suffering from moderate to severe blindness [2]. According to the 1998 World Health Report, 19.34 million people are blind bilaterally (less than 3/60 in the better eye) as a result of age-related cataracts. This accounted for 43% of all blindness cases [3]. The cataract is becoming worse by the day. Recent cases of cataract increased by 43.6%, with nuclear cataracts accounting for 23.1%, Posterior Subcapsular Cataracts (PSC) for 13.1%, and cortical cataracts for 22%, and cataract surgery was done only for 26.8%. Besides that, all types of cataract surgery have increased in recent years. Studies show that there are more female patients compared to males. This includes nuclear and cortical cataracts and cataract surgery (*p* = 0.02–0.05). In addition, it is more common in the nonwhite community (*p* = 0.001) [4].

Cataracts develop as a result of aging and the use of crystalline lenses. Many interdependent elements, including the lens' microscopic structure and chemical content, preserve the lens' transparency and optical homogeneity. A progressive deposit occurs in the lens where a yellow-brown pigment is seen which increases with aging. This also reduces the transmission of light into the eyes. The symptoms of cataract basically depend on the types of cataracts, the lifestyle of a person, and also his visual requirements. Intracapsular and extracapsular cataract extractions are the two terms used interchangeably. Intracapsular extraction entails removing the entire lens while keeping the capsule intact. In the developed world, this approach is hardly used for treatment. It is still popular in underdeveloped countries since it requires fewer expensive and sophisticated instruments. It does not need a highly stable electricity supply. Besides that, it can be performed within a short training period. Another method is extracapsular extraction. The nucleus of the lens is removed in one piece; a relatively large incision is required. Cataract disease can be detected using transfer learning-based intelligent methods and ocular image datasets. Preliminary cataract detection and prevention may help to minimize the rate of blindness. This approach is cheap and efficient, which is the main motivation of this study.

In recent years, better cataract surgery has been created than in the previous 20 years. Around 85-90% of patients who experience cataract surgery will have 6/12 (20/40 or 0.5) best-corrected vision in patients with no ocular comorbidity such as macular degeneration, diabetic retinopathy, or glaucoma [5]. When the patient is in the early stages of cataract, their response to refractive glasses is typically good. Patients should be admitted to the hospital for surgical cataract removal and intraocular lens implantation if outpatient treatment with refractive glasses and pupillary dilation fails to improve their vision [6].

### 1.1. Related Work

We looked at current journals and publications to better understand the problem and discussed viable solutions for improving the accuracy of our deep learning model. To compare our efforts, we used an existing dataset and looked at their model. Preprocessing, feature extraction, feature selection, and classifier or mode are the four key elements of the cataract classification method. A study says that image processing techniques can be used for detecting cataract in eyes through analyzing fundus images. A group of researchers used two methods to analyze fundus images. One is the Novel Angular Binary Pattern (NABP), and another approach was the Kernel-Based Convolutional Neural Networks, and their proposed method accuracy was 0.9739 [7].

Recently, proposed residual networks (ResNets) exhibited cutting-edge performance in the ILSVRC2015 classification challenge, allowing the training of extraordinarily deep networks with more than 1000 layers. For picture classification, the ResNet model is employed. An article entitled “Eye Disease Detection using RESNET” shows 0.0925 accuracies in their method where the optimum epoch value was 30 [8]. Pratap and Kokil did more research and collected data from various resources. They had 800 images and they used DL. They achieved an accuracy of 92.91% [9]. There could be a variation in the results in a larger dataset. In addition, in this article, the results of several imaging modalities used for cataract disease grading were compared. Basic information on cataracts was presented, including how to tell the difference between normal and cataract vision, as well as the many forms of cataract illness [10]. Sertkaya et al. suggested a study to investigate retinal illnesses using convolutional neural networks and coherent optical pictures. Their respective methods were AlexNet, LeNet, and Vgg16. In the Vgg16 and AlexNet architectures, they achieved good results. Here, the overall accuracy was 82.9% [11]. Gosh et al. suggested a study that used CNN and a dataset that consisted of glaucoma, retinal disease, and normal eye cataracts. Their accuracy was judged to be 82%, which is acceptable by CNN standards [12].

In the research, a machine learning-based algorithm that supports vector machines was used to identify cataracts. This method divides the entire photo into 17 pieces in this system, with each portion feeding into the Support Vector Machine (SVM) algorithm. This method has an accuracy of 87.52%. However, it cannot identify partial cataracts [13]. An active shape model trained on over 5000 images was used in a recent study and achieved 95.00 percent accuracy [14]. In the case of high-dimension feature maps, SVM is not an appropriate option. Hossain et al. authored a paper entitled “Automatic Detection of Eye Cataract using Deep Convolution Neural Networks.” In his work, he used Deep Convolution Neural Networks, and the module was ResNet50 to detect cataracts and noncataract fundus. Their overall validation accuracy was 97.38% where their training accuracy was nearly 100% [15]. Li et al. introduced a ResNet-based discrete state transition (DST) system. Their accuracy in cataract detection performance was 94.00%, and they solved the vanishing gradient issues. The recommended DC-NN design overcomes the gradient concerns by using the residual connection technique. It also removes the need for picture preprocessing and can transmit high-dimensional characteristics [16]. Recent research by Ahmed et al. on cataract using CNN with VGG-19 has acquired an overall 97.47% accuracy where the precision was 97.47% and the loss was 5.27% [17].

Different authors have proposed various models, and they have achieved different accuracy levels. The proposed model in this research shows better results compared with previous work, so this research is novel. The major contribution of this paper is to detect cataract disease using transfer learning-based intelligent methods. This paper presents the comparison of the performances of four distinct deep learning models, namely, DenseNet121, Xception, InceptionV3, and InceptionResNetV2, on training, validation, and test datasets for cataract disease detection. Various approaches and hyperparameters have been employed to implement those models in this research to accurately distinguish normal and cataract photos. After that, the best model has been found for the further classification of normal and cataract images.

An introduction has been provided in Section 1. Section 2 discusses the methodology, and Section 3 presents the results and analysis.  Section 4 contains the conclusion.

## 2. Methodology

This section describes specific processes that are followed and maintained in order to conduct tests on the project for cataract disease detection. The workflow of the best model selection is shown in Figure 1(a). Figure 1(a) shows how the model predicts the disease from raw data through the training and validation stages by selecting various hyperparameters. This methodology segment will give a quick overview of each of the blocks listed below and their importance in this research.

The workflow of the cataract or normal image detection is depicted in Figure 1(b). To diagnose, the image is fitted to the best trained model after preprocessing, and the model notifies whether the image has cataract disease or not.

### 2.1. Dataset

The dataset employed in this suggested system consists of 1088 fundus pictures. Shanggong Medical Technology Co., Ltd. collected the pictures from various hospitals and medical institutions around China. The Ocular Disease Intelligent Recognition (ODIR) database is a structured ophthalmic database including 5000 patients' ages, color fundus images of their right and left eyes, and diagnostic keywords given by doctors [18]. The dataset is made up of actual patient data. From the previously mentioned datasets, we solely utilized cataracts and ordinary fundus pictures for our purposes.

### 2.2. Preprocessing

The proposed system dataset combines photographs of normal, diabetes, glaucoma, cataract, pathological myopia, hypertension, age-related macular degeneration, and other diseases/abnormalities. As a result, we have separated all fundus photographs except cataract and ordinary fundus photographs in the first phase. Labels were used to filter the data. Because they were obtained with different cameras, experimental fundus pictures had varying image sizes. As a result, we used OpenCV to resize the picture to 224 × 224 pixels. The dataset is next loaded and converted into an array format for training purposes using the NumPy library.

### 2.3. Overview of the Proposed Model

The following are explanations of the models utilized in this research study, as well as their block diagrams to clarify the motivation behind using transfer learning models.

*InceptionV3*: InceptionV3 [19] outperforms earlier inception designs in terms of computing efficiency. Inception modules are the fundamental components of an inception model. Through dimensionality reduction with layered 1 × 1 convolution, the inception module enables fast computing and deeper networks. The modules were designed to address a variety of problems, including computational cost and overfitting. The inception module's main notion is to run several filters of varied sizes in parallel in preference to series. The inception modules' networks contain an additional 1 × 1 convolution layer, previously the 3 × 3 and 5 × 5 convolution layers, making the method computationally cheap and reliable.

In this experiment, we used a pretrained InceptionV3 model. InceptionV3 begins with weight = “imagenet,” including_top = False, input_shape = (224,224,3); these starting values, and GlobalAveragePooling2D layers, are shown in Figure 2(a). A dense block follows, followed by a BatchNormalization () layer. There are 512 hidden layers in the dense block and a “relu,” a rectified linear activation function, which is a linear operation that produces directly when given a positive insert. Or else, a value of 0 will be returned. It is the default option, and it yields the best results. The “relu” function is used to solve the vanishing gradient problem, allowing models to learn quickly and with higher accuracy. The logistic function sigmoid activation function is the final layer. It takes any real value as an input and outputs a number between 0 and 1. The compressed form of InceptionV3, which was used in this study, is shown in Figure 2(a).

*Xception*: “extreme inception” is what Xception [20] stands for. Xception was first shown in 2016. There are 36 layers in the Xception model, excluding the completely linked layers at the conclusion. Xception has depth-wise separable layers as well as “shortcuts” that combine the production of individual layers with the output of preceding layers. Unlike InceptionV3, Xception packages compress data into a few lumps. It independently maps the spatial linkages for each yield channel, then performs 1 × 1 depth-wise convolutions to capture cross-channel interactions. In the categorization of the ImageNet dataset, Xception surpasses Inception v3. A pretrained Xception model was used in our research. Because large-scale datasets for cataract disease diagnosis are lacking, a pretrained model is employed.  Figure 2(b) shows how the Xception model works for our research.

This network, likewise, addresses DenseNet121. The vanishing gradient problem is caused by network depth. To guarantee the maximum flow of information between levels, all the layers' connection designs are used. Each layer receives input from the earlier layers in this configuration and transmits its intrinsic feature maps to the next layers. To transmit data from one layer to the next, the feature maps are concatenated at each layer. The number of parameters has been considerably decreased since this network architecture eliminates the need to remember redundant data. Due to its many layer connection features, it is also effective at retaining information [21]. DenseNet121 is a more efficient convolutional neural network than DenseNet, which performs deep analysis and provides simple output. Without the initial layer, each layer in DenseNet121 is linked to the previous levels. One layer's output is utilized as an input for the next layer. Each layer has a direct link to the next. The DenseNet121 model for our research is depicted in Figure 2(c).

### 2.4. Overview of the Best Model

*InceptionResNetV2*: InceptionResNetV2 was established by merging the two most popular deep convolutional neural networks, Inception [22] and ResNet [23], and using batch-normalization for the conventional layers rather than summations. The leftover modules are specifically utilized to enable a higher quantity of Inception blocks and, as a consequence, a deeper system. As previously stated, the utmost apparent difficulty related to extremely deep networks is the training stage. That may be handled via residual connections. While a huge number of filters are used in a system, the residual is scaled down as an effective way to deal with the training difficulty. When the number of strainers surpasses 1000, the residual variations encounter instability, and the network cannot be trained. As a result, the residual aids are scaled in network training stabilization. The compressed form of InceptionResNetV2, which was used in this study, is manifested in Figure 3.

*Sigmoid function*: the sigmoid function [4] is a numerical measure that has the feature of transferring any actual value to a range between 0 and 1, shaped like the letter “S.” The logistic function is another name for the sigmoid function. The sigmoid function's equation is

(1) $$\begin{array}{c} X=\frac{1}{1+e^{-Y}}. \end{array}$$

The main advantage of the sigmoid function is that it exists between two points, 0 and 1. As a consequence, it is very effective in models where we need to anticipate probability as an output. We chose this function since the chance of something occurring is only between 0 and 1.

*ReLU*: the rectified linear activation unit (ReLU) [24] is one of the few milestones in the deep learning revolution. It is basic yet far superior to previous activation functions such as sigmoid. The following is an example of how to write this operation.

(2) $$\begin{array}{c} f\left(\text{input}\right)=\max\left(0,\text{input}\right). \end{array}$$

According to the equation, the greatest value between zero and the input value is the output of ReLU. When the input value is negative, the output is equal to zero, and when the input value is positive, the output is equal to the input value. This may be written in simple terms as follows:

if input>0:

return input

else:

return 0

### 2.5. Evaluation Metrics

In this study, the following performance matrices were used to evaluate the performance of several models:

*Accuracy*: accuracy is one criterion for evaluating classification models. Casually, validity relates to our model's percentage of true projections. The following formula is used to calculate binary classification accuracy in terms of pros and cons:

(3) $$\begin{array}{c} \text{Accuracy}=\frac{\text{TP}+\text{TN}}{\text{TP}+\text{TN}+\text{FP}+\text{FN}}. \end{array}$$

*Recall*: divide the number of True Positives (TP) by the number of True Positives and False Negatives (FN) to get the recall. On the other hand, the number of positive predictions divided by the number of positive class values in the test data equals the number of positive forecasts divided by the number of positive class values in the test data. It is also known as the “True Positive Rate” or “Sensitivity.”

(4) $$\begin{array}{c} \text{Sensitivity}/\text{Recall}=\frac{\text{TP}}{\text{TP}+\text{FN}}. \end{array}$$

*Precision*: precision is calculated by dividing the total number of True Positives and False Positives (FP) by the number of True Positives. To put it another way, it is the total number of positive predictions divided by the total number of expected positive class values. Positive Predictive Value is another name for it.

(5) $$\begin{array}{c} \text{Precision}=\frac{\text{TP}}{\text{TP}+\text{FP}}. \end{array}$$

*Specificity*: the percentage of true negatives that are predicted to be negative is known as specificity. As a result, a tiny number of true negatives will be projected as positives, leading to false positives. This fraction is also known as the “false positive rate.” The sum of specificity and false positive rate is always equal to one.

(6) $$\begin{array}{c} \text{Specificity}=\frac{\text{TN}}{\text{TN}+\text{FP}}. \end{array}$$

*F1 score*: the F1 score is a common measure for classification tasks, and it is useful when accuracy and recall are both important. The *F* score, sometimes recognized as the F1 score, assesses a model's accuracy on a specified dataset. It is used to evaluate binary classification algorithms that sort things into positive and negative categories. True predictions, whether positive or negative, are always great. These are the goals we want to achieve using our methodology. False predictions, on the other hand, should be avoided. We strive to minimize these occurrences to a bare minimum. The *F* score is a method for determining a model's accuracy and recall. This is calculated as follows:

(7) $$\begin{array}{c} \text{F}1\text{ score}=\frac{2\times \text{Precision}\times \text{Recall}}{\text{Precision}+\text{Recall}}. \end{array}$$

*Confusion matrix*: it is the most useful diagram for deciphering the model's performance details. Important predictive measures such as recall, specificity, accuracy, and precision are calculated using confusion matrices. Confusion matrices are beneficial because they make comparing values like True Negatives, False Negative (FN), True Positives, and False Positives straightforward. This was crucial for our study, since we needed to assure accuracy as well as recall. Our goal was to detect infected pictures with minimal or no misclassification, which we were able to do using the InceptionResnetV2 model. Consequently, we were able to estimate the overall model performance in terms of specificity and sensitivity/recall.

## 3. Result Analysis

This section explains how four different pretrained models, such as DenseNet121, InceptionV3, Xception, and InceptionResNetV2, were used to detect cataract illness. First, the dataset was downloaded from Kaggle and divided into training (80%) and validation (20%) sets, as shown in Table 1. We used 588 cataract pictures and 500 normal images in this sample, where all the images have been resized to 224 × 224.

Then, utilizing various hyperparameters, we developed and compiled those four pretrained models.  Table 2 demonstrates that the initial learning rate is retained at 1*e*-5, the batch size is 32, the maximum epoch is 15, and the optimizer is the “Adam” optimizer when building the pretrained models. The optimizer maintains a decay of 1*e*-3/epoch and a loss function of “binary cross-entropy.” Finally, all the models have been run on Colab, and the execution environment is kept as “GPU.”

Figure 4(a) and Figure 3(b) represent the accuracy and loss graph of the DenseNet121 model, respectively. When the DenseNet121 model has been fitted to the dataset, at the first epoch, the training accuracy is 87.47% and the loss is 35.86%. But the validation accuracy is very poor (48.62%) and the loss is also very high (12582%), which indicates that the model initially learns very poorly. As the number of epochs increases, training and validation accuracy both increase, and the loss function also starts to decrease. At epoch 10, the DenseNet121 model found its highest validation accuracy, which is 95.41%. At that time, validation loss was 23.13%, training accuracy was 97.70%, and training loss was 6.54%. After epoch 10, the model overfits the data, which is why there is a high fluctuation in the graph after epoch 10. Therefore, an early stop method has been used to stop the model from overfitting.

The accuracy and loss graph of the Xception model are shown in Figures 5(a) and 5(b), respectively. When the Xception model is fitted to the dataset, the training accuracy is 94.83 percent at the first epoch, while the loss is 13.62 percent. However, the validation accuracy is a little low (61.47%), and the loss is 59.61%, indicating that the model learns quite better compared to the DenseNet121 model at first. The training accuracy grows as the number of epochs increases, but the validation accuracy graph always fluctuates. On the other hand, both the loss functions start to decrease. The model achieved its best validation accuracy of 97.71 percent at epoch 7. Validation error was 7.02 percent, training accuracy was 98.97 percent, and training error was 3.33 percent at the moment. After epoch 7, this model also overfits the data, resulting in a significant level of fluctuation in the graph. An early halting approach was applied to prevent the model from overfitting.

The InceptionV3 model's accuracy and loss graph are illustrated in Figures 6(a) and 6(b), respectively. The training accuracy is 88.74 percent at the first epoch when the InceptionV3 model is fitted to the dataset, whereas the loss is 45.32 percent. However, the validation accuracy is 53.67 percent, but the validation loss is very high (1260.18 percent). As the number of epochs grows, so does the training and validation accuracy, while the loss function decreases. The InceptionV3 model achieved its highest validation accuracy of 97.71 percent at epoch 6. At that time, the validation error was 12.23 percent, the training accuracy was 98.05 percent, and the training error was 5.02 percent. This model also overfits the data after epoch 6, resulting in a substantial amount of fluctuation in the graph. An early stopping method was also used here to prevent the model from overfitting.

Finally, the InceptionResNetV2 model is fitted to the dataset. Figures 7(a) and 7(b) show that, at epoch 1, this model's training accuracy and loss were 91.03% and 26.10%, while the validation accuracy and loss were very poor (53.21% and 2364407.03%, respectively). The training accuracy grows gradually along with the number of epochs. At first, the validation accuracy was fluctuating, but after some epochs, it was quite stable. The model achieved its highest validation accuracy (98.17%) at epoch 11, while the validation loss is 6.22%, the training accuracy is 99.54%, and the training loss is 1.94%. After that, the accuracy graph again fell due to overfitting.

The Model Check Point has been used to save the best trained model. The best trained DenseNet121 model was evaluated on the test dataset after completing 5 epochs, and Table 3 reveals that the model achieves 95.41 percent testing accuracy and 23.13 percent testing loss. It can also be seen that the DenseNet121 model has a sensitivity of 92.30 percent and a specificity of 98.42 percent. This model also detects normal images with precision, recall, and F1 score of 98 percent, 92 percent, and 95 percent, respectively, and cataract images with precision, recall, and an F1 score of 93 percent, 98 percent, and 96 percent, respectively. Table 3 also shows that, on the test dataset, the best-trained Xception model achieves 97.71 percent testing accuracy and 7.19 percent testing loss. The model also achieves a sensitivity of 97.92 percent and a specificity of 97.54 percent. However, this model has a precision, recall, and F1 score of 97 percent, 98 percent, and 96 percent for recognizing normal photos, respectively, and 93 percent, 98 percent, and 97 percent for detecting cataract images, respectively. The InceptionV3 model also does quite well at detecting cataract disease, with an accuracy and loss of 97.71 percent and 12.23 percent on the test dataset, respectively. It has a sensitivity of 95.04% and a specificity of 100%. The InceptionV3 model has stopped training after 6 epochs due to a higher risk of overfitting, and its precision, recall, and F1 score on normal images are 100 percent, 95 percent, and 97 percent, respectively, while its precision, recall, and F1 score on cataract images are 96 percent, 100 percent, and 98 percent, respectively. Finally, according to its performance results, the InceptionResNetV2 model's test accuracy is 98.17 percent, loss is 6.22 percent, sensitivity is 96.55 percent, and specificity is 100 percent. In the detection of normal images, this model achieves 100 percent, 97 percent, and 98 percent precision, recall, and F1 score, respectively, and 96 percent, 100 percent, and 98 percent precision, recall, and F1 score in the detection of real photos, respectively. When these four models are examined, it becomes clear that the InceptionResNetV2 model has the highest accuracy when compared to the others.

In recognizing normal and cataract photos, Figure 8 displays True Positive, True Negative, False Positive, and False Negative cases. According to the results, the DenseNet121 model predicts normal images 92% accurately as “normal,” while incorrectly predicting 8% of normal images as “cataract.” The figure also shows that the model predicts 98% of cataract photos that are truly “cataract,” while 2% of photos are wrongly predicted as “normal.”

The Xception model properly predicts normal images 94% of the time as “normal,” while mistakenly identifying normal images 6% of the time as “cataract,” as seen in Figure 9. It also demonstrates that the program correctly predicts 98 percent of cataract photos as “cataract,” but only 2% of cataract photos as “normal.”

Figure 10 shows that the InceptionV3 model properly predicts normal images 96 percent of the time as “normal,” while wrongly identifying normal photos 4% of the time as “cataract.” The image also demonstrates that the model correctly identifies 100 percent of cataract photos as “cataract.”

Figure 11 shows that the InceptionResNetV2 model properly predicts normal images 97% of the time as “normal,” while wrongly predicting normal photos 3% of the time as “cataract.” The image also indicates that the program correctly classifies 100 percent of cataract photos as “cataract.”

Our work is compared with all the previous research work mentioned in Related Work. In that case, we can conclude that, by using the same dataset, the VGG-19 model got the highest accuracy of 97.47% to date. Both AlexNet and LeNet got the overall accuracy of 82.9%. The SVM algorithm got 95% accuracy after being trained into 5000 images. The ResNet50 model got an accuracy of 97.38% in the classification of cataract and noncataract fundus. On the other hand, our proposed best trained InceptionResNetV2 model achieved the training accuracy of 99.54% and validation or testing accuracy of 98.17% by using only 588 normal images and 500 cataract images which reached the new state-of-the-art. Hence, this research work is novel.

## 4. Conclusion

Pretrained models such as InceptionV3, InceptionResNetV2, Xception, and Densenet121 are used in this article to offer an automated cataract diagnosis method. The InceptionResNetV2 model, which can now identify cataract disease with a test accuracy of 98.17%, a sensitivity of 97%, and a specificity of 100%, has effectively reached the new state-of-the-art. Given the preceding reasoning, an automated cataract diagnostic system would be highly useful in poor countries with insufficient numbers of qualified ophthalmologists to treat patients. Such approaches would make healthcare more accessible, reduce time and screening costs for both the patient and the ophthalmologist, and enable early diagnosis. In the future, we can focus on improving the accuracy of the model by using a larger and more complex dataset. We can also try to apply various image processing methods so that the model can learn the image pattern more accurately and give better accuracy more efficiently. We can also build a website for easy access by all people worldwide.

## Figures and Tables

**Figure 1:** (a) Workflow of the best model selection. (b) Workflow of the cataract or normal image detection.

**Figure 2:** Block diagram of InceptionV3, Xception, and DenseNet121.

**Figure 3:** Block diagram of InceptionResNetV2.

**Figure 4:** (a) Accuracy graph of DenseNet121 model and (b) loss graph of DenseNet121 model.

**Figure 5:** (a) Accuracy graph of Xception model and (b) loss graph of Xception model.

**Figure 6:** (a) Accuracy graph of InceptionV3 model and (b) loss graph of InceptionV3 model.

**Figure 7:** (a) Accuracy graph of InceptionResNetV2 and (b) loss graph of InceptionResNetV2.

**Figure 8:** Confusion matrix for DenseNet121.

**Figure 9:** Confusion matrix for Xception.

**Figure 10:** Confusion matrix for InceptionV3.

**Figure 11:** Confusion matrix for InceptionResNetV2.

**Table 1:** Split the dataset into training, validation, and test sets.

Dataset	Number of images
Cataract	588
Normal	500

**Table 2:** Parameters used for compiling various models.

Parameters	Value
Initial learning rate	1*e*-3
Decay	(1*e*-3)/epoch
Batch size	32
Shuffling	Each epoch
Optimizer	Adam
Loss	Binary cross-entropy
Epoch	5
Execution environment	GPU

**Table 3:** Performance score of DensNet121, Xception, InceptionV3, and InceptionResNetV2.

Model	Dataset	Accuracy	Loss	Sensitivity	Specificity	Images	Precision	Recall	F1 score
DenseNet121	Test	0.9541	0.2313	0.9230	0.9842	Normal	0.98	0.92	0.95
						Cataract	0.93	0.98	0.96
Xception	Test	0.9771	0.0719	0.9792	0.9754	Normal	0.97	0.98	0.97
						Cataract	0.98	0.98	0.98
InceptionV3	Test	0.9771	0.1223	0.9504	1.00	Normal	1.00	0.95	0.97
						Cataract	0.96	1.00	0.98
InceptionResNetV2	Test	0.9817	0.0622	0.9655	1.00	Normal	1.00	0.97	0.98
						Cataract	0.96	1.00	0.98

## Data Availability

The data utilized to support these research findings is accessible online at https://www.kaggle.com/andrewmvd/ocular-disease-recognition-odir5k.
